# HOXB13, a Target of DNMT3B, Is Methylated at an Upstream CpG Island, and Functions as a Tumor Suppressor in Primary Colorectal Tumors

**DOI:** 10.1371/journal.pone.0010338

**Published:** 2010-04-29

**Authors:** Kalpana Ghoshal, Tasneem Motiwala, Rainer Claus, Pearlly Yan, Huban Kutay, Jharna Datta, Sarmila Majumder, Shoumei Bai, Arnab Majumder, Tim Huang, Christoph Plass, Samson T. Jacob

**Affiliations:** 1 Department of Molecular and Cellular Biochemistry, Ohio State University, Columbus, Ohio, United States of America; 2 Comprehensive Cancer Center, Ohio State University, Columbus, Ohio, United States of America; 3 Division of Epigenomics and Cancer Risk Factors, German Cancer Research Center, Heidelberg, Germany; 4 Department of Molecular Virology, Immunology and Medical Genetics, Ohio State University, Columbus, Ohio, United States of America; University of Birmingham, United Kingdom

## Abstract

**Background:**

A hallmark of cancer cells is hypermethylation of CpG islands (CGIs), which probably arises from upregulation of one or more DNA methyltransferases. The purpose of this study was to identify the targets of DNMT3B, an essential DNA methyltransferase in mammals, in colon cancer.

**Methodology/Principal Findings:**

Chromatin immunoprecipitation with DNMT3B specific antibody followed by CGI microarray identified genes with or without CGIs, repeat elements and genomic contigs in RKO cells. ChIP-Chop analysis showed that the majority of the target genes including *P16*, *DCC, DISC1, SLIT1, CAVEOLIN1, GNA11*, *TBX5, TBX18, HOXB13* and some histone variants, that harbor CGI in their promoters, were methylated in multiple colon cancer cell lines but not in normal colon epithelial cells. Further, these genes were reactivated in RKO cells after treatment with 5-aza-2′-deoxycytidine, a DNA hypomethylating agent. COBRA showed that the CGIs encompassing the promoter and/or coding region of *DCC, TBX5, TBX18, SLIT1* were methylated in primary colorectal tumors but not in matching normal colon tissues whereas *GNA11* was methylated in both. MassARRAY analysis demonstrated that the CGI located ∼4.5 kb upstream of HOXB13 +1 site was tumor-specifically hypermethylated in primary colorectal cancers and cancer cell lines. *HOXB13* upstream CGI was partially hypomethylated in *DNMT1^−/−^* HCT cells but was almost methylation free in cells lacking both DNMT1 and DNMT3B. Analysis of tumor suppressor properties of two aberrantly methylated transcription factors, HOXB13 and TBX18, revealed that both inhibited growth and clonogenic survival of colon cancer cells *in vitro*, but only HOXB13 abolished tumor growth in *nude* mice.

**Conclusions/Significance:**

This is the first report that identifies several important tumor suppressors and transcription factors as direct DNMT3B targets in colon cancer and as potential biomarkers for this cancer. Further, this study shows that methylation at an upstream CGI of *HOXB13* is unique to colon cancer.

## Introduction

Symmetrical methylation of DNA at position 5 of cytosine within a CpG dinucleotide is a major epigenetic modification (∼5% of the total cytosine in the mammalian genome) although a small amount of 5-hydroxymethylcytosine (5hmC) generated from 5-meC by a methylcytosine dioxygenase has recently been detected in certain cell types [1]–[3]. Very recently it has been shown that cytosine methylation at nonCpG sites, although rare, is involved in gene silencing in mammals [4]. DNA methylation is essential for mammalian development. DNA hypermethylation suppresses spurious promoters located within the repeat elements and proviruses in mammalian genome whereas hypomethylation induces genomic instability [5], [6]. DNA methylation is also involved in the regulation of genomic imprinting, inactivation of the silent X chromosome in females and expression of certain tissue specific genes [1], [6]. In humans, alterations in genomic methylation patterns are linked to imprinting disorders and other human diseases including cancer [7]–[9].

Although CpG is usually underrepresented in much of the genome, short (500–2000 bp long) CpG regions, designated CpG islands (CGI), are predominantly located in the proximal promoter regions of almost 50% of the mammalian genes. These regions are usually methylation free in normal cells with the exception of imprinted alleles and genes on the inactive X chromosome. Recent high throughput genome wide DNA methylation analysis identified many more CGIs located distal to promoters that are tissue-specifically methylated [5]. Furthermore, methylation also occurs in the coding regions of active genes and reversible DNA methylation can regulate gene expression in response to stimuli such as estrogen treatment and membrane depolarization [6].

DNA methylation in mammalian cells is established and maintained by DNA (cytosine-5) methyltransferases (DNMTs). Methylation is initiated by highly homologous DNMT3A and DNMT3B that prefer unmethylated DNA as the substrate [1], [10]. DNA methylation is heritably propagated by DNMT1 that prefers hemimethylated DNA as substrate. All three DNMTs are essential for development in mammals [11], [12]. Among these three enzymes, DNMT3B is directly linked to different diseases. For example, mutation of the DNMT3B gene causes immunodeficiency, centromeric instability and facial anomalies (ICF) syndrome, a rare human disorder due to alteration in the methylation of minor satellite repeats [13] and genes regulating immune function and neuronal development [14]. Thus, DNMT3B deficiency in these patients cannot be compensated by other DNMTs. Studies in mutant mice have shown that DNMT3A and DNMT3B methylate distinct as well as overlapping regions of the genome [12]. For example, DNMT3A2 catalyzes methylation of imprinted genes in germ cells whereas tandem repeat elements are methylated by both DNMT3A and DNMT3B [2]. DNMT3B has also been linked to type 2 diabetes by regulating mitochondrial DNA copy numbers through fatty acid-induced non-CpG methylation of PGC-1α [4]. Emerging studies have shown that a variety of cofactors specifically target DNMTs to distinct chromosomal regions in vivo [15], as these enzymes demonstrate specificity only towards CpG base pairs *in vitro* [2]. Gene silencing by DNMTs occurs predominantly by recruitment of repressors that include methyl CpG binding proteins (MBDs) and co-repressors such as histone deacetylases (HDAC) and histone methyltransferases (HMT), resulting in distortion of local chromatin structure [3], [9], [16].

Hypermethylation of CpG islands (CGIs) is a common epigenetic event in almost all malignancies [7], [9]. Upregulation of DNMT3B is also a characteristic of many cancer cells [17]. For example, in sporadic breast carcinoma, 30% of the patients showed increased expression of DNMT3B compared to minimal increase (3–5%) in DNMT1 and DNMT3A [18]. Significantly higher expression of DNMT3B was observed in acute myeloid leukemia compared to normal myeloid cells [19]. DNMT3B overexpression was associated with high tumor grade and CIMP (CpG island methylator phenotype) in colon cancer [17]. Furthermore, depletion of DNMT3B, but not DNMT3A, induced apoptosis specifically in human cancer cells [20]. It has also been reported that upregulation of DNMT3B is more dramatic and more frequent than DNMT1 and DNMT3A in cancers including bladder and colon [21]. Studies in a mouse model have shown that the overexpression of Dnmt3b but not Dnmt3a promoted colon tumorigenesis in Apc^Min/+^ mice [22]. These observations suggest that DNMT3B may play a causal role in tumorigenesis.

Different groups have identified methylation targets using different techniques [14], [22], in the present study we have identified direct DNMT3B target genes in colon cancer cells by performing chromatin immunoprecipitation followed by CpG island microarray analysis (ChIP-on-chip). Many DNMT3B targets are embedded in CpG islands and some are known tumor suppressors. We also report the methylation status of some of these genes with potential growth suppressor properties in primary colorectal tumors and colon cancer cell lines. Further, we examined tumor suppressive characteristics of two important transcription factors, HOXB13 and TBX18, in colon cancer cells.

## Methods

### Mice

Nude mice were purchased from Jackson laboratory. All mice were housed, handled, and euthanized in accordance with federal and institutional guidelines under the supervision of the Ohio State University Institutional Animal Care and Use Committee. All animals used in this study were handled in strict accordance with good animal practice as defined by the relevant national and/or local animal welfare bodies.

### Cell culture, treatment with 5-aza-2′-deoxy-cytidine (decitabine) and isolation of DNA

Human colon cancer cell lines (RKO, HCT116, SW480, SW837, Colo205, CaCo2 and DLD1b) and normal colon cell line (CCD841) were obtained from ATCC and grown in media as suggested by ATCC. RKO and HCT116 cells were treated with decitabine (0.1 to 5 µM) for 24–120 hours. The wild type, *DNMT1^−/−^, DNMT3B^−/−^* and DKO (*DNMT1−/− DNMT3B^−/−^*) cells (a generous gift from Bert Vogelstein) were cultured as described [23].

### Western blot analysis

Affinity purified antibodies against DNMT3A and DNMT3B were used for western blot analysis as described [24], [25]. Anti-Flag antibody was from Sigma.

### Primary Human Tumors

The tumor samples were obtained from patients at James Cancer Hospital (The Ohio State University). Complete pathologic classification is available for all tumor samples studied. All tissues used for this study were part of an institutional review board-approved protocol at the Ohio State University College of Medicine.

### ChIP on Chip assay

Chromatin immunoprecipitation (ChIP) assay was performed as described [26] with some modifications. ChIP was performed on formaldehyde cross-linked chromatin (DNA fragmented to ∼600 bp to 3000 bp by sonication) from 10^8^ RKO cells with antibody against DNMT3B [26], [27]. The anti-DNMT3B antibodies raised in our laboratory do not cross react with each other or with DNMT1 [28]. We used affinity purified DNMT3B antibodies to pull down DNA from formaldehyde cross-linked chromatin prepared from RKO cells. The chromatin was cleared with pre-immune IgG and protein A beads. The precipitated DNA was dissolved in RIPA buffer and subjected to a second round of immunoprecipitation with the same antibody to minimize pull down of false positive targets. This DNA was then separated on an agarose gel and DNA from 0.5 to 3 kb in size was purified by using Gel Extraction kit (Qiagen), labeled with Cy5-labeled dNTP and hybridized to a CpG island library coated on glass slides [29], [30]. The same amount of input DNA and DNA precipitated with preimmune-IgG) was used as control. We selected only those genes for sequence analysis where the signal in ChIP DNA was ≥2 fold compared to the control rabbit IgG signal. MIAME complaint data has been submitted to Geo database (accession number GSE18929).

### Sequence analysis of clones

The construction of CpG island library has been described earlier [29]. The clones pulled own by DNMT3B antibodies were picked up from the CpG island library and sequenced in an automated sequencer.

### RT-PCR and real-time RT-PCR analysis

RNA was isolated using guanidinium thiocyanate-acid phenol method, treated with DNase 1 to remove residual DNA, if any, and reverse transcribed using random hexamers following standard protocol. Real time RT-PCR was done using SYBR Green technology following published protocol [27], [31]. RT-PCR primers will be available upon request.

### ChIP-CHOP analysis was performed as described [32]

Primer sequences are provided in the **Table S1**.

### COBRA (Combined bisulfite-restriction analysis)

**COBRA** of genomic DNA was performed as described [33], [34]. CGIs different genes were amplified with primers specific for bisulfite converted DNA where unmethylated cytosines are converted to uracils. Primers were designed using Methprimer software (http://www.urogene.org/methprimer/index1.html). Primer sequences are provided in the **Table S1**.

### Quantitative DNA methylation analysis of HOXB13 CGI by MassARRAY

DNA methylation analyses were carried out using the EpiTYPER application (Sequenom, San Diego) as described [35]. Briefly, genomic DNA was isolated, subjected to integrity control and subjected to bisulfite treatment. Regions of interest were amplified using primers for bisulfite treated DNA (primer sequences available upon request), amplified DNA was transcribed *in vitro* and cleaved using RNAse A. The molecular weight of the resulting fragments indicative of the DNA methylation state was analyzed using matrix-assisted laser desorption ionization time-of-flight (MALDI-TOF) mass spectrometry. DNA methylation standards (0, 20, 40, 60, 80 and 100%) were used to control for PCR amplification bias. Equation fitting algorithms based on the R statistical computing environment were used for data correction. Display of methylation results as heat maps and unsupervised clustering were performed using the Multiple Experimental Viewer software (http://www.tm4.org/mev.html).

### Cloning of HOXB13 and TBX18 cDNA and generation of RKO and HCT116 cell lines overexpressing these proteins

cDNA derived from total RNA from normal human colon (Clontech) was amplified with primers specific for *HOXB13* and *TBX18* coding region and cloned into pcDNA-3XFlag (Sigma). The authenticity of the cDNAs was confirmed by sequencing. The Flag-tagged cDNAs were then cloned into pBabe-puro and infectious retroviruses were generated in phoenix cells. Stable cell lines (RKO, HCT116 or DLD1b) overexpressing HOXB13 or TBX18 were generated by infecting these cells with the recombinant retroviruses and selected with puromycin.

### Clonogenic survival was performed as described [36]

### Cell growth was measured by MTT assay as described[37]

### Tumor growth in nude mice was performed as described [38]

### HOXB13 promoter activity assay

*HOXB13* promoter regions spanning −1.2 kb to +0.2 kb and −5.2 kb to +0.2 kb with respect to transcription start site (TSS) were amplified from lymphocyte DNA using Accuprime polymerase, confirmed by sequencing, and cloned into pGL3 basic (firefly luciferase vector). These promoter reporter plasmids along with pRLTK (renilla luciferase vector) were transfected into RKO cells and luciferase activity was measured using Dual luciferase assay kit (Promega).

## Results

### ChIP on Chip analysis identified DNMT3B target genes in RKO, a colon cancer cell line

Aberrant DNA methylation is prevalent in colorectal carcinogenesis [39]–[41]. To identify hypermethylated genes in colon cancer (RKO) cells we performed ChIP with anti-DNMT3B followed by CpG island (CGI) microarray. We selected DNMT3B because its expression is significantly higher than DNMT3A and DNMT1 in RKO cells (**Figure 1A**) and it appears to play a causal role in colon tumorigenesis [22]. The specificity of the affinity purified DNMT3B antibody was confirmed by using extracts from DNMT3B *null* HCT cells. A major (∼98/96 kDa) polypeptide was detected by this antibody in RKO cells, in the wild type and *DNMT1^−/−^* HCT cells. That these polypeptides are different variants of DNMT3B was confirmed by the inability of the antibody to detect any protein in *DNMT3B^−/−^* and DKO (*DNMT1^−/−^ DNMT3B^−/^*) cells. A few very minor polypeptides detected in cells expressing DNMT3B are probably its isoforms because it is known that DNMT3B exhibits different spliced variants [42]. To reduce nonspecific pull down, ChIP was performed twice with the same antibody and the precipitated DNA was resolved on an agarose gel to elute DNA of smaller sizes (0.5 to 3 kb) as probe for CpG island microarray (see Methods for detail) (**Figure 1B**).

**Figure 1:** Expression of DNMT3B is higher in RKO cells. **A.** Western blot analysis of whole cell extracts from RKO and HCT (wild type and mutant) cells with antibodies specific for DNMTs. Affinity purified antibodies against DNMT3B were used for immunoblotting. **B.** Real-time RT-PCR analysis of DNMTs in RKO cells was performed using SYBR Green method. Data are mean of triplicate assays. Single and double asterisks denote p values ≤0.05 and ≤0.01, respectively. **C.** Ethidium bromide staining of DNA immunoprecipitated by DNMT3B antibody and input DNA that were used for CpG island microarray analysis.

Next, we sequenced only those pulled-down genes that were at least 2 fold enriched in ChIP DNA compared to that pulled down by control rabbit IgG. The microarray data has been submitted to Geo database and it is MIAME complaint (accession number GSE18929). We classified these genes into four groups, i) genes with CpG island (CGI) but without repeat elements, ii) genes without CGI and repeat elements, iii) repeat elements, and iv) genomic contigs associated with repeat elements (**Table 1** **and Table S2**). Among the genes with CGIs, there are some known tumor suppressors, such as *P16/MTS1, DDC, PGRMC1, CAVEOLIN1* and some disease susceptibility genes such as *DISC1* (disrupted in Schizophrenia 1) [43], *TBX5* (Congenital heart failure or Holt-Oram syndrome) [44] (**Table 1**). We also identified a few novel genes such as *TBX18, DGKI, SLIT1* and *GNA11* as DNMT3B targets.

**Table 1:** Methylted DNMT3B Target Genes in RKO cells identified by ChIP on Chip.

Accession #	Gene name	Gene symbol
	GROUP I: Genes harboring CpG island without repeat elements	
NM_018662	disrupted in schizophrenia 1	DISC1
NM_003522	histone cluster 1, H2bf	HIST1H2BF
NM_001080508	T-box 18	TBX18
NM_001753	Caveolin-1	CAVEOLIN1
NM_004717	diacylglycerol kinase iota	DGKI
U26727	P16INK4/MTS1	CDKN2A
NM_021951	doublesex and mab-3 related transcription factor 1	DMRT1
NM_003692	transmembrane protein with EGF-like and two follistatin-like domains 1	TMEFF1
NM_003061	Slit-1	SLIT1
NM_018362	lin-7 homolog C (C. elegans)	LIN7C
AF532858	Nogo-66 receptor homolog-1	NGRH1/RTN4RL2
BC031869	M.m. C.elegans ceh-10 homeo domain containing homolog	Chx10
NM_181486	T-box 5	TBX5
NM_006361	homeodomain protein HOXB13	HOXB13
NM_005215	colorectal tumor suppressor	DCC
NM_002067	guanine nucleotide-binding regulatory protein, alpha-11	GNA11
NM_006667	progesterone receptor membrane component 1	PGRMC1
NM_024784.3	zinc finger and BTB domain containing 3	ZBTB3
	GROUP II: Genes with no CGIs or repeat elements	
AY210419	CUB and sushi multiple domains 3	CSMD3

Association of DNMT3B to the target genes and their methylation status was determined by ChIP-CHOP assay. Formaldehyde-cross-linked chromatin from RKO cells was immunoprecipitated with anti-DNMT3B or pre-immune IgG. DNA pulled down was divided into three aliquots, which were either undigested or digested with *Hpa* II, *Msp* I and subjected to PCR with primers specific for CGIs of different genes that harbor *Hpa* II/*Msp* I sites. PCR products were resolved by agarose gel electrophoresis. Generation of PCR product in *Hpa* II digested DNA indicates methylation.

To confirm the association of DNMT3B with some of its putative target genes, we amplified their promoter regions from a different batch of chromatin immunoprecipitated DNA. We performed ChIP-CHOP analysis to determine methylation status of the target DNA. For this assay, the immunoprecipated DNA was divided into three identical aliquots for mock-digestion, digestion with *Hpa* II (methylation sensitive enzyme) or *Msp* I (methylation insensitive enzyme) (see **Figure 2A** for a schematic diagram). The digested DNA was then used to amplify the promoter of interest using primers that encompass one or more *Hpa* II/*Msp* I sites. Amplification of the promoter region from the mock-digested DNA indicates that the gene of interest is a target of DNMT3B whereas generation of *Hpa* II resistant PCR product demonstrates that the gene is methylated. PCR products are not obtained from *Msp* I digested DNA since *Msp* I digestion is not sensitive to methylation. Thus, ChIP-CHOP assay not only reveals association of a gene with a certain protein but also identifies the methylation status of the associated promoter at *Hpa* II sites. The data presented in **Figure 2B** demonstrated that some of the DNMT3B target genes such as *P16*, *TBX5, TBX18, GNA11, DMRT1, HOXB13, CAVEOLIN1, PGRMC1, DCC, DGKi, CDH26, LIN7C, ZBTB3, DISC1* and the histone H2B variant (*H2Bf*) are methylated in RKO cells. Notably, *TBX-18, HOXB13, DMRT1, DISC1, H2Bf and LIN7C* CGIs are partially methylated in RKO cells at least at the *Hpa* II sites (as demonstrated by increased PCR product in mock-digested DNA than in *Hpa* II cleaved DNA) and DNMT3B is associated with these CGIs irrespective of their methylation status. In contrast, DNMT3B is predominantly associated with methylated CGIs of *P16, TBX5, DCC* and *PGRMC1*. None of these target genes could be amplified from chromatin immunoprecipitated with control rabbit IgG (data shown for only TBX5) (Fig. 2B) demonstrating that these are specific DNMT3B targets. Lack of amplification of *GAPDH* promoter, a house keeping gene, from RKO genomic DNA indicates that GAPDH CGI is methylation free and *Hpa* II digestion was complete. GAPDH was not pulled down by DNMT3B (data not shown).

**Figure 2:** ChIP-CHOP assay to demonstrate association of DNMT3A and DNMT3B with the selected target genes. **A.** Schematic diagram of ChIP-CHOP assay. **B.** Formaldehyde-cross-linked chromatin from RKO cells was immunoprecipitated with anti-DNMT3B or pre-immune IgG. DNAs pulled down were divided into three aliquots, which were either undigested or digested with *Hpa* II, *Msp* I and subjected to PCR with primers specific for CGIs of different genes that harbor *Hpa* II/*Msp* I sites. PCR products were resolved by agarose gel electrophoresis. Generation of PCR product in *Hpa* II digested DNA indicates methylation. U, H and M indicate PCR products obtained in mock-, *Hpa* II- digested and *Msp* I-digested DNA, respectively. Lack of PCR product with *Msp* I digested DNA confirmed complete digestion. **C.** Activation of several DNMT3B target genes in RKO cells after treatment with decitabine. RKO cells were treated with the drug for the indicate time periods. RNA from these cells was subjected to RT-PCR with gene-specific primers. Three hundred ng of cDNA for the test gene and 1 ng of cDNA were used for 18S rRNA.

Next, we tested methylation status of a few genes in other colon cancer cell lines (DLD1b, HCT116, SW480, CACo2, COLO205, SW837) by digestion of their genomic DNA with *Hpa* II/*Msp* I followed by PCR with gene specific primers. While *TBX5* and *DCC* are methylated in all cell lines, other genes (*TBX18, DGKI, PGRMC1, LIN7C* and *HOXB13*) are differentially methylated (**Table S3**). It is noteworthy that none of these genes are methylated in normal colon epithelial cells CCD841.

### Treatment of RKO cells with decitabine resulted in activation of the methylated genes

To determine whether methylation of some of the DNMT3B target genes indeed suppressed their expression in RKO cells, we treated these cells with the commonly used DNA hypomethylating agent, 5-aza-2′-deoxycytidine. RNA isolated from untreated and the inhibitor (1 and 2.5 µM) treated RKO cells harvested at 24, 48 or 72 hours was subjected to RT-PCR analysis with gene specific primers. *TBX18, DCC* and *CAVEOLIN 1* were re-expressed in RKO cells treated with 1 and 2.5 µM decitabine as early as 24 hr and their expression persisted up to 72 hr (**Figure 2B**). In contrast, *SLIT1* was induced at a very low level under these conditions whereas HOXB13 was reactivated only after exposure to the drug for 72 hr. On the contrary, *GNA11* was expressed at high level in RKO cells indicating that the methylation of CGI located in intron 1 of this gene did not affect its expression.

### CGIs of DNMT3B target genes are methylated in human primary colorectal tumors

Next, we extended our study to analyze the methylation status of a selected group of genes (*DCC, TBX18, TBX5, SLIT1* and *GNA11*) in several primary human colorectal tumors and matching normal colon tissues by COBRA. The methylation status of these genes in a few pairs is presented in **Figure 3**. The CGI spanning promoter/exon 1 of *DCC* was methylated at *Taq* I site in 8 out of 10 tumors as demonstrated by almost complete digestion with *Taq* I whereas it was methylated in matching normal colon tissues only in sample #8 and #10 (**Figure 3** **.i**). Similarly, CGI of *TBX18* was methylated at the *Bst*U I site in 6 out of 7 tumors without significant methylation in matching normals (**Figure 3** **.ii**). *TBX5* encodes 4 transcript variants that are generated by alternate transcription initiation sites and alternative splicing. We analyzed methylation status of CGIs spanning the promoter/exon 1 of variants 1 and 3 (TBX5L) and variant 4 (TBX5S) (**Figure 3** **.iii**). Interestingly, CGI of TBX5L was methylated at *Taq* I sites both in normal colon tissues and tumors but methylation was more pronounced in 3 out of 5 tumors (#1, 4 & 6) than in the matching normals. In contrast, CGI of TBX5S was specifically methylated in tumors in 5 out of 6 samples at the *Bst*U I site. Thus, two CGIs located in close proximity demonstrated differential methylation status in the same sample at least with respect to *Taq* I and *Bst*U I sites. CGI spanning promoter/exon 1 of *SLIT1* was tumor-specifically methylated at the *Taq* I site in 5 out of 10 samples analyzed (**Figure 3** **.iv**). Notably CGI located in the intron of *GNA11* was completely methylated both in normals and tumors as demonstrated by complete digestion of the PCR product with *Bst*U I (**Figure 3** **.v**). Methylation at this intronic CGI did not silence *GNA11* as demonstrated by its robust expression in RKO cells (**Figure 2c**). Complete bisulfite conversion was demonstrated by digestion of the amplicons with methylation insensitive *Mse* I or *Tsp*509 I (data not shown). These COBRA data showed that some of DNMT3B targets were hypermethylated in primary colorectal tumors albeit at different levels. However, we did not observe methylation of CGI located in the promoter as well as exon 1 region of the *HOXB13* gene in primary colon cancer by COBRA (data not shown).

**Figure 3:** Analysis of methylation status of CGI of selected genes by COBRA in primary human colorectal tumors. Location of the CGI of each gene as appeared in UCSC genome browser is depicted in the accompanied schematic diagrams. Bisulfite converted genomic DNA was amplified with gene specific primers followed by digestion with a methylation sensitive enzyme *Taq* I or *Bst*U I. T and N denote tumor and matching normal, respectively. Sample numbers shown in red identify tumors with gene-specific methylation.

### CGI located 4.5 kb upstream of *HOXB13* Transcription start site (TSS) is hypermethylated in colorectal tumors

Although COBRA did not reveal methylation of CGI located in the promoter and exon 1 region, *HOXB13* gene was reactivated after treatment with decitabine (**Figure 2C**). This observation suggested that methylation of a CGI located at a different region of the gene or specific CpGs within the promoter region might regulate its expression in colon cancer cells or tissues. BLAT analysis identified two CGIs in human *HOXB13* gene, one in the promoter/exon1 and the other ∼4.5 kb upstream of transcription start site (TSS) (**Figure 4A**). We, therefore, analyzed methylation status of CpGs spanning the promoter and upstream CGI (**Figure 4B** **, and Tables S4 and S5**) in primary colorectal tumors and in cell lines by MassARRAY because in this mass spectrometry based assay methylation status of CpGs can be estimated quantitatively. It is evident from the HEAT map that methylation at the upstream CGI is higher in tumors than in normals (**Figure 4C** **.i**). Quantification of the results showed that overall methylation density at the upstream CGIs was significantly higher (P = 0.02) in tumors compared to the normals (**Figure 4C** **.ii**). In contrast, CGI in the promoter region was essentially methylation free (**Figure 4C** **.i**), which correlated with the COBRA data (data not shown). MassARRAY analysis of colon cancer cell lines revealed hypermethylation at the upstream CGI in HCT, CaCo2 and RKO cells whereas relatively low level methylation was detected in RWPE and SW837 cells. Notably, CCD841, a normal colon epithelial cell line, was essentially unmethylated. Selective methylation of the upstream CGI but not the one located in the immediate upstream promoter region occurs in colon cancer cells probably due to distinct chromatin structure that is accessible to DNMTs.

**Figure 4:** Methylation of the CpGs spanning upstream and promoter regions of *HOXB13* gene in primary colorectal tumors and colon cancer cell lines by MassARRAY. **A** and **B. Potential methylatable CpGs in these regions are shown after bisulfite conversion.** CpGs sequenced by MassARRAY are boxed and numbered. It is notable that this technique provides average methylation status of CpGs that are in close proximity (numbered together as 1, 2 etc). Gray bars indicate samples that could not be sequenced. **C.i.** HEAT map of methylation profile of CpGs located within upstream CGI and promoter (TSS) region. The same amplicon of methylation density ranging from 0 to 100% was used to generate standard curve. **C.ii.** Box plot of quantitative analysis of methylation density in the upstream CGI and promoter regions in primary colorectal tumors and normals. Significance was assessed by Welch test (adaptation of t test, parametric, unequal variance, one-tailed). **D. Upstream region (−5.4 kb) activates** ***HOXB13*** **promoter activity in colon cancer cells.** *HOXB13* promoter regions (−1.2 kb and −5.4 kb) cloned into pGL3 basic vector (RLU1) were transfected into HCT116 cells along with internal control pRLTK (RLU2), followed by treatment with 10 nM estradiol (E) in phenol red free medium containing 5% charcoal stripped serum for different time periods. **E.** Only the upstream CGI is methylated in HCT cells, which undergoes site-specific and global demethylation by DNMT1 alone and both DNMT1, DNMT3B, respectively. **i**) MassARRAY, **ii**) real-time RT-PCR analysis of HOXB13, and iii) RT-PCR analysis of ERα and GAPDH.

To investigate the role of the upstream CGI in *HOXB13* expression we generated luciferase reporter constructs harboring −5.4 kb to +0.2 kb and −1.2 kb to +0.2 kb regions, respectively into pGL3basic vector and compared their ability to modulate firefly luciferase activity at 36 and 48 hr post transfection in HCT116 cells, because these cells can be transfected with high efficiency. The luciferase activity driven by −5.4 kb promoter was at least 2 fold higher than that contributed by −1.2 kb region (**Figure 4D**). Promoterless pGL3basic showed minimal activity (data not shown). Since *HOXB13* is an estrogen responsive gene [45], we also measured activity of these two promoter regions by treating cells with estrogen 24 hr post-transfection with estradiol that increased the activity of both promoters at 12 and 24 hrs (**Figure 4D**). Taken together, these results demonstrated that the upstream promoter region of *HOXB13* gene stimulated promoter activity but did not contribute to estrogen responsiveness.

To identify the DNA methyltransferase (DNMT) that catalyzes methylation of HOXB13, we measured its methylation status in the wild type and mutant HCT cell lines lacking *DNMT1*, *DNMT3B* or both. Massarray analysis showed that the upstream CGI is heavily methylated in the wild type and *DNMT3B−/−* cells but is significantly hypomethylated at certain CpGs in *DNMT1−/−* cells and almost completely in double knock out (DKO) cells (**Figure 4E** **and Tables S4 and S5**). These results indicate that although DNMT1 alone can methylate certain CpGs, its cooperation with *DNMT3B* is required for efficient methylation of the upstream CGI. Notably, promoter CGI is not methylated in any of these 4 cell lines. Surprisingly, HOXB13 expression is upregulated only in *DNMT1−/−* cells compared to the wild type cells (**Figure 4E**). Significant downregulation of ERα (**Figure 4E**), an activator of HOXB13 [45] probably accounts for HOXB13 suppression in *DNMT3B−/−* and DKO cells. Increase in HOXB13 expression in *DNMT1−/−* cells suggests that methylation at certain CpGs in the upstream CGI suppresses HOXB13 expression. Thus, the upstream CGI probably functions as an enhancer and its methylation partially suppresses but does not silence HOXB13 expression.

### Ectopic expression of TBX18 and HOXB13 inhibits growth, clonogenic survival and anchorage independent growth of colon cancer cells

We next explored the anti-tumorigenic properties of TBX18 and HOXB13 in colon cancer cells. TBX18, a member of T-box family of transcription factor, is expressed in the segmented somites and in the limb bud [46]. TBX18 knock out mice die immediately after birth due to severe defects in organs deriving from the lateral sclerotome [47]. In contrast, ubiquitously expressed HOXB13 is a member of homeobox super family involved in establishing cell fate during embryonic development and maintaining differentiation state in adults [48], [49]. HOXB13 is upregulated in many solid tumors including cancers of the endometrium, cervix, ovary and prostate whereas it is down regulated in renal cell carcinoma, melanoma and colon cancer [45]. To study the potential role of HOXB13 and TBX18 in modulating tumorigenic property of colon cancer cells we expressed these proteins using retroviral vector (pBabe) in the nonexpressing colon cancer cell lines RKO and DLD1b. Ectopic expression of the proteins was measured in puromycin-selected cells by Western blot analysis with anti-Flag antibody (**Figure 5A**). The growth rates of TBX18 and HOXB13 expressing versus nonexpressing cells were assessed by MTT assay. Overexpression of these proteins resulted in a significant decrease in the growth rate of the cells compared to vector starting from day 1 in both cell lines (**Figure 5B**), which correlated with dramatic reduction in replication potential in RKO cells expressing TBX18 or HOXB13 compared to vector transfected cells (**Figure 5C**). Similarly, clonogenic survival of RKO cells expressing these transcription factors was significantly reduced (**Figure 5D**). Ectopic expression of HOXB13 and TBX18 in another nonexpressing cell line, DLD1b inhibited these properties (data not shown). Together, these results demonstrated that TBX18 and HOXB13 severely compromised tumorigenic potential of colon cancer cells in vitro.

**Figure 5:** HOXB13 and TBX18 demonstrate anti-tumorignic property in colon cancer cells in vitro. **A.** Western blot analysis of cell extracts prepared from RKO cells expressing Flag-tagged HOXB13 or TBX18. Analysis of cell growth by MTT assay (**B**), replication potential by ^3^H_1_-thymidine incorporation (**C**), clonogenic survival (**D**) of RKO cells (pool and a clone selected at random). Each assay was performed in triplicate. Single and double asterisks denote p values ≤0.05 and ≤0.01, respectively.

### HOXB13 but not TBX18 inhibits growth of colon cancer cells in *nude* mice

We next investigated whether HOXB13 and TBX18 expression could inhibit *ex vivo* growth of colon cancer cells. For this purpose, RKO cells expressing either HOXB13 or TBX18 and vector transfected cells were injected into the flanks of *nude* mice. Mice were monitored for tumor growth every week and tumor size was measured. Tumor growth was visible as early as one week in mice injected with the control and TBX18 expressing cells. In contrast, the tumor was not detectable in most of the animals injected with HOXB13 expressing cells (**Figure 6A**). At the end of the experiment, the mice were sacrificed, tumors were removed and their weights and volumes were determined. Notably, HOXB13 expressing cells could not form tumors in majority of animals (**Figure 6B, C**). These cells formed only two visible tumors in mice. Surprisingly, no significant change in tumor growth in RKO cells expressing TBX18 was observed. Western blot analysis with anti-Flag antibody to detect ectopic TBX18 showed that the tumors developed nude mice expressed TBX18 (**Figure 6D**) suggesting that lack of inhibition of tumor growth in nude mice was not due to loss of TBX18 expression. It is likely that some host factor(s) in the tumor microenvironment antagonizes the tumor suppressor function of TBX18 in nude mice. Similar results were observed in HCT116 and DLD1b cells (data no shown). Thus, HOXB13 functions as a tumor suppressor in colon cancer cells both in vitro and *ex vivo*.

**Figure 6:** HOXB13 but not TBX18 inhibited ability of RKO cells to form tumor in nude mice. One million cells in PBS (100 µl) were injected into the flanks of nude mice and tumor size was monitored every week using a caliper. After 25 days tumors were excised and their weights were documented. **A.** Time course of the progression of tumor growth. **B.** Photograph of the tumors developed by vector-transfected, HoxB13 or TBX18 expressing cells. **C.** Tumor weight at the time of sacrifice. D. Western blot analysis of ectopic TBX-18 in the tumors T1 to T4 (shown in A) with anti-Flag antibody.

## Discussion

It is now well established that hypermethylation is a common mechanism for silencing tumor suppressor genes in cancer cells. Because re-expression of these genes upon demethylation was perceived to be an alternate strategy for cancer therapy, considerable effort has been expended to identify novel tumor suppressor genes in specific cancer types that are silenced by methylation. Clinical trials of Vidaza and Dacogen against different cancers underscore the significance of epigenetic therapy in cancer [50], [51]. Further, differentially methylated genes could be potential biomarkers for colorectal cancer. Indeed, recent studies have shown that some of the hypermethylated genes could be detected in the stool of colon cancer patients [41], [52].

DNA methyltransferases, expressed at relatively low levels in somatic cells, are frequently upregulated in cancer cells. Gain of function studies have shown that Dnmt3b but not Dnmt3a promotes colon tumorigenesis in APC^Min/+^ mice by inducing de novo methylation of multiple genes harboring CpG islands [22]. It, therefore, becomes important to identify the targets of DNMT3B in colon cancer cells to understand its function in tumorigenesis. A recent study has used expression profiling to identify its targets in colon cancer cell lines [53]. To our knowledge, the present study is the first report on the identification of direct DNMT3B targets in colon cancer cells using ChIP-on-chip with antibodies that are specific for DNMT3B. The targets identified include not only well known tumor suppressors such as *P16/INK4A, DCC, CAVEOLIN1, PGRMC1* but also novel genes like *TBX18, TBX5, SLIT1, DGKI*. Activation of some of these genes after treatment with demethylating agents confirmed that methylation indeed silenced their expression in colon cancer cells. DNMT1 and DNMT3B function co-operatively to methylate and silence many tumor suppressor genes in colon cancer cells [23]. It is, therefore, conceivable that both enzymes could act in concert to alter methylation status of the target genes, as observed in HOXB13 upstream CGI (Figure 4E).

An important observation is that a validated set of genes (*TBX5, DCC, DGKI, CDH26, HOXB13, CAVEOLIN1, PGRMC1, GNA11, TBX18, ZBTB3 and DMRT1*) are indeed associated with DNMT3B and that they are methylated in more than one colon cancer cell line relative to normal colon epithelial cells (CCD841). Among these, only *DCC* [54] and *CAVEOLIN1* [55] have recently been reported to be methylated in colorectal carcinoma. DMRT1 is methylated in gastric cancer [56] whereas HOXB13 is methylated in melanoma [57], renal cancer [58] and breast cancer [45]. Further, analysis of a subset of these genes (*DCC, TBX18, TBX5, SLIT1*) in primary colon cancer revealed tumor-specific methylation. Recently several investigators have identified genes methylated in colorectal cancer some of which were also detected in the stool of colorectal cancer patients [41]. Different etiology, genetic background and the techniques used probably account for the identification of distinct methylated genes [59]. Cluster analysis demonstrated that tumors with dense methylation at the upstream CGI of HOXB13 gene clustered together (**Figure S1**). It would be of interest to analyze a large cohort of colorectal tumors to determine whether methylation of HOXB13 occurs in specific type of tumors and this epigenetic modification can be used as a diagnostic or prognostic marker for colorectal cancer.

HOXB13 belongs to the homeobox family of transcription factors. It is a unique developmentally regulated protein that is up- or down-regulated depending upon the cellular context. While it is upregulated in ovarian [60] and endometrial cancers [61] where it functions as a tumor promoter, its expression is suppressed in malignant melanoma [57], renal [58], prostate [62], colorectal [63] and breast [45] cancer. *HOXB13* is methylated in malignant melanoma, renal and breast cancer in the CGIs spanning the immediate upstream promoter and exon 1. Surprisingly, this region is essentially methylation free in normal colon and colorectal tumors (Figure 4). Methylation at an upstream CGI located ∼4.5 kb upstream of the HOXB13 transcription start site in primary colorectal tumors and colon cancer cell lines suggests that chromatin structure of this region acquires a unique conformation accessible to DNMTs. C/EBPα is another transcription factor that is tumor-specifically methylated at an upsteam CGI in lung [64] and head and neck cancer [65]. Recent high throughput analysis has identified many more genes that are methylated at far upstream CGIs and even in coding regions [6]. The upstream CGI of *HOXB13* appears to contribute to its promoter activity in colon cancer cells and harbors several conserved cis-regulatory elements some of which encompass CpG dinucleotides. It is, therefore, likely that methylation of this region is involved in modulating expression of *HOXB13* and that this mechanism is unique to colon cancer cells. It would be of interest to examine whether HOXB13 knockout mice are susceptible to colon tumorigenesis spontaneously, after crossing with Apc/^Min+^, *Mlh1^−/−^* mice or upon exposure to carcinogens. Similarly, identification of HOXB13 target genes in colon epithelial cells is likely to elucidate the mechanism of its tumor suppressor function. Generation of immunoprecipitation grade antibody for HOXB13 will help us to answer this question. Studies along these lines are in progress.

## Supporting Information

Table S1 List of primers (ChIP-CHOP, COBRA, RT-PCR, cDNA cloning and promoter regions) used in the present study. COBRA primers were designed using Methprimer database (http://www.urogene.org/methprimer/index1.html).
(0.11 MB DOC)

Table S2 Chromatin from RKO cells were immunoprecipitated with affinity purified Dnmt3B antibodies or mock-immunoprecipitated. Precipitated DNA ranging in size from 0.6 to 3 kb were subjected to CpG island microarrary. The chromatin was cleared with pre-immune IgG and protein A beads. The precipitated DNA was dissolved in RIPA buffer and subjected to a second round of immunoprecipitation with the same antibody to minimize pull down of false positive targets. This DNA was then separated on an agarose gel and DNA from 0.5 to 3 kb in size was purified by using Gel Extraction kit (Qiagen), labeled with Cy5-labeled dNTP and hybridized to a CpG island library coated on glass slides. The same amount of input DNA and mock-immunoprecipitated DNA (with rabbit preimmune-IgG) was used as control. We selected only those genes for further analysis where the signal in ChIP DNA was greater than 2 fold compared to the control rabbit IgG signal.
(0.16 MB DOC)

Table S3 Genomic DNA from different colon cancer and normal colon epithelial (CCD841) cells were digested with Hpa II, Msp I or mock-digested and an aliquot (100 ng) of DNA from each was subjected to PCR with primers specific for CGI of each gene followed by separation of the PCR products on an agarose gel. The gene was codiered to be methylated if PCR product was generated in the Hpa II digested DNA but not in Msp I digested DNA.
(0.08 MB DOC)

Table S4 MassARRAY data of upstream CGI of HOXB13 gene in primary colon cancer and matching colon tissues and colon cell lines (normal and cancer). Methylation at each CpGs was determined based on a standard curve generated using methylation density ranging from 0% to 100% of the amplicon.
(0.02 MB XLS)

Table S5 MassARRAY data of promoter CGI of HOXB13 gene in primary colon cancer and matching colon tissues and colon cell lines (normal and cancer). Methylation at each CpGs was determined based on a standard curve generated using methylation density ranging from 0% to 100% of the amplicon.
(0.03 MB XLS)

Figure S1 Unsupervised clustering of human primary colorectal tumors (T) and matching normal colon tissues (N) methylation based on methylation density at upstream CGI of HOXB13 as determined by MassARRAY.
(9.75 MB TIF)
